# Multiple Impacts of Urban Built and Natural Environment on Lung Cancer Incidence: A Case Study in Bengbu

**DOI:** 10.1155/2023/4876404

**Published:** 2023-02-04

**Authors:** Kangkang Gu, Yuwei Li, Xianjie Jia, Chengrong Liu

**Affiliations:** ^1^School of Architecture & Planning, Anhui Jianzhu University, Hefei, Anhui, China; ^2^Research Center of Urbanization Development in Anhui Province, Hefei, Anhui, China; ^3^Department of Epidemiology and Statistics, School of Public Health, Bengbu Medical College, Bengbu 233000, China

## Abstract

Tumours are the main disease affecting the health of the Chinese population, and lung cancer is the malignancy with the highest incidence. Hence, the need to study and analyse the population of lung cancer incidence in order to effectively control and prevent it. In this research, we discuss the demographic characteristics of lung cancer incidence population of 2014 to 2020 from the perspective of multiple urban environmental factors, taking Bengbu city in the Huaihe River Basin of China as the research area, analyse the correlation between environmental indicators and lung cancer incidence population through the Spearman's rank correlation assessment model, and analyse the interaction between the influence factors of a geographic detector to analyse the influence of urban environmental factors. The results showed the followings: (1) The distribution characteristics of lung cancer incidence population were mainly geriatric population and spatially mainly fell in the old urban area of the study area, and the population distribution had clustered characteristics. (2) Through Spearman's rank correlation analysis, the land use, road traffic, spatial form, service facilities, and the open space of green space of the urban-built environment as well as the natural environment are all correlated with the incidence of lung cancer. (3) Factor detection and interaction analysis revealed a greater effect of spring and winter on lung cancer prevalence. In addition, the road intersection density and the distance to industrial are the most important potential influencing factors, and the interaction of any two factors will increase the risk of lung cancer.

## 1. Introduction

Environmental and health issues are gradually becoming an important aspect of current national and international research, especially for the exploration of the prevention of chronic noncommunicable diseases, while cancer has been a major cause of global health problems, and due to the lagging nature of cancer, the crude incidence rate and the age-standardised incidence rate (asir) of cancer in 2016 were 293.91 per 100,000 and 186.46 per 100,000, respectively, and the crude mortality rate was 174.55 per 100,000 and the age-standardised mortality rate (as) was 105.19 per 100,000 according to the National Cancer Centre Journal. Lung cancer has the highest incidence and mortality among cancers, making research on the lung cancer population an important current public health issue. In China, lung cancer has been the cancer with the highest incidence and mortality rates [1], and the Chinese Health Statistical Yearbook also shows that mortality from respiratory diseases such as pneumonia and pneumoconiosis among residents of large cities is increasing every year [2]. In this context, the prevention and control of lung cancer disease have attracted attention, and how to prevent the occurrence of lung cancer and reduce the risk factors brought about by the environment is the focus of current research.

In recent years, there has been an increasing number of studies on the factors influencing lung cancer in the population both at home and abroad. Smoking and passive smoking, genetic factors, air pollution, and dietary exposure are considered to be important risk factors for lung cancer. The urban environment has many factors affecting the population of lung cancer and the mechanisms of influence are complex [3]. A large number of studies have demonstrated that the incidence of respiratory diseases is significantly correlated with the concentration and characteristics of airborne particulate matter [4]. The elevated concentrations of atmospheric particulate matter in the city will cause decreased lung function of residents, thereby resulting in severe respiratory diseases; moreover, a large number of automobile exhaust emissions caused by high-density road traffic [5], the heavy pollutants from industrial diffusion [6], and the cooking fumes of restaurants will all contribute to the increase in particle concentration [7], causing public health problems. Meanwhile, urban form and spatial structure also constitute the important reasons for the increase in urban PM concentrations [8, 9]. Generally speaking, the higher building density and floor-area ratio of a city will cause the worse ventilation conditions and the higher incidence of respiratory system diseases [10].

In addition, the existing studies have shown that vegetation allocation also has a significant impact on neighborhood space, shrubs have a positive effect on the respiratory system [11], the increase of green coverage is beneficial to the reduction in the concentrations of particulate matters [12], and a certain scale of park green space can reduce PM_2.5_ [13]. Therefore, higher regional vegetation allocation can reduce the incidence of lung cancer and promote respiratory health. According to the foreign studies of Hankey et al., the health benefits brought by the increased physical activity of residents in communities with high walking rates can properly offset the adverse effects of air pollution [14]. Proper physical activity can promote physical and mental health and reduce the risk of lung cancer.

In general, the research on respiratory health mainly includes macroscopic [15, 16] and microscopic [17] studies, and it has been found that buildings, transportation, and land use of the urban-built environment have a certain influence on the population of people who develop lung cancer. Nevertheless, there are few studies on diverse urban environments and even fewer studies on its mechanism. Therefore, based on a case study on a certain district, Bengbu City, Huaihe River Basin, the incidence of lung cancer was analysed and explored, the distribution and influencing mechanism of lung cancer among urban residents were probed, and the correlation between urban spatial factors and the incidence of lung cancer, as well as the environmental factors and characteristics significantly related to the distribution of patients were clarified. Furthermore, some suggestions on the optimization of planning control and urban design were put forward, so as to provide theoretical basis and practical direction for reducing the risk of respiratory diseases of urban residents and creating a healthy urban living space.

## 2. Study Area and Data Source

### 2.1. Study Area

The study area is located in the old city of Bengbu, Anhui Province, China. Bengbu is an important industrial city in China and is located in the south of the Huaihe River Basin in China, Huaihe River Basin, one of the most densely populated basins in China, with prominent diversity and complexity of population and is particularly seriously affected by urban-spatial factors. In 2020, the total area of Bengbu City were 5,952 square kilometers, with a registered population of 3.863 million and an urbanization rate of 58.6%. And the 7th census shows that in 2020, 18.03% of Bengbu's population will be over 60-years-old, and the aging rate is accelerating. According to international regulations, people aged 65 years and over are the elderly, taking into account the legal retirement age and other practical circumstances in China, and persons with 60 years of age and over are selected as the criteria for older persons. As an important industrial city, the study area is located in the old urban area in the west of Bengbu City, with a registered population of 360,000, and it is also the administrative region with the largest population in Bengbu City, characterized by high population density and rapid urbanization, so it is suitable for the urban environment and population health research. The study area consisted of 12 blocks numbered YH01-12, which were divided into 2,744 spatial units by 100 m grids, and the outliers are excluded (Figure 1). The study area is located in the midlatitude region, and the winter average temperature is 1°C and is vulnerable to the cold air temperature.

### 2.2. Data Source

The relevant data on people who developed lung cancer were obtained from all inpatients diagnosed with lung cancer by Bengbu Health Commission from 2014 to 2020, and all information about lung cancer patients, including age, gender, and residential address, were extracted. Inpatients whose home addresses and workplaces were not in the study area were excluded from the inpatient data, giving a final total of 449 cases. The number of residents of the study area was derived from the official bulletin of the Bengbu National Bureau of Statistics.

The land-use data and the built-environment data for the study area in the environmental data were obtained from the Anhui Urban & Rural Planning and Design Institute, and the data contained the main uses of each land in the study area in 2019 (Figure 2(a)), which included the road system, green space and river, residential land, and industrial land according to urban land classification, including the base area and floor number of each building. The data for commercial and bus stops are derived from the Baidu Map Open Platform's point of interest (POI) data, which has the characteristics of a large sample size, wide coverage, and detailed spatial resolution, which makes the spatial analysis more comprehensive, objective, and in-depth. Using Landsat 8 remote sensing data provided by the United States Geological Survey (USGS) and the code LC81210372019023LGN00, the natural environment data of the Bengbu Ecological Environment Agency and the geospatial data cloud were obtained, and the air pollution index is based on the 2014–2020 average of Bengbu's state-controlled environmental monitoring sites.

### 2.3. Establish an Indicator System

By constructing environmental factor evaluation indicators from the acquired environmental indicator data, a system of urban environmental impact-factor indicators such as land use, road traffic, space form, green space and open space, air pollution and temperature, and service facilities was established to analyse the impact of the natural and built environment on the incidence of lung cancer (Table 1). The incidence rate of lung cancer is calculated as follows:

(1) $$\begin{array}{c} Incidence=\frac{NC}{NP}\times 100\%\text{.} \end{array}$$

*NC* is the number of lung cancer patients in the unit and *NP* is the total population in the unit.

After excluding the abnormal value, we analysed the index that might affect the incidence of lung cancer, and the correlation index was *P* < 0.05, which had a statistical significance.

## 3. Statistical Analysis

### 3.1. Spearman's Rank Correlation

Spearman's correlation coefficient for ranked data is a statistical method used to evaluate the correlation between two variables. The most remarkable characteristic of Spearman's correlation is that it does not need to consider the sample size or the overall distribution of variables [18], and it is fast and robust [19]. Therefore, we use Spearman's rank correlation to analyse the correlation between lung cancer incidence population and different environmental factors in cities, in which lung cancer incidence and environmental factors are normalized, the range of the values is [0, 1], to balance the dimension gap of data, so that different data are counted under the same conditions, and the calculation formula is as follows:

(2) $$\begin{array}{c} r_{s}=1-\frac{6\sum_{i=1}^{n}d_{i}^{2}}{n\left(n^{2}-1\right)}\text{.} \end{array}$$

In the formula, *r*_*s*_ is the Spearman's correlation coefficient; the range of the values is [−1, 1], the bigger the absolute value is, the stronger the correlation is; *n* is the number of lung cancer disease areas; and *i* = 1…*n. d*_*i*_ represents the rank difference between the values of dependent lung cancer disease and independent environmental factors.

### 3.2. Geographical Detector

Geographical detector is a spatial analysis model used to detect the relationship between a geographical attribute and its explanatory factors and can be used to show whether the relationship between the indicator factors has a significant difference in the spatial distribution of the impact, measured by *q* statistics, with a value ranged [0, 1] [20, 21]. If stratified on the population of lung cancer incidence, higher values indicate a higher degree of spatial heterogeneity in respiratory disease, and if stratified on the value of lung cancer disease according to the influence indicator, higher values indicate a higher degree of explanation of respiratory disease by that influence indicator, in addition to the absence of spatial heterogeneity when the *q* value is 0. This study used geographical detector software for factor interaction detection and *k*-means clustering of the continuous detection factor values in SPSS. The formula is as follows:

(3) $$\begin{array}{c} q=1-\frac{\sum_{h=1}^{L}N_{h}\sigma_{h}^{2}}{N\sigma^{2}}\\ =1-\frac{SSW}{SST}\text{.} \end{array}$$

SSW=∑_*h*=1_^*L*^*N*_*h*_*σ*_*h*_^2^, SST=*Nσ*^2^.

The study area is divided into strata, *h* = 1, ... *L*, and *N*_*h*_ and *N* represent the layer *h* and the number of units in the study area, respectively. *σ*^2^ represents the variance of lung cancer population, *σ*_*h*_ represents the variance of index in the layer, and SSW and SST are the sum of Within sum of squares and total sum of squares, respectively.

## 4. Results

### 4.1. Distribution Characteristics of Lung Cancer Incidence

During the period from 2014 to 2020, a total of 449 cases of lung cancer were collected in the study area of Bengbu City, and the basic characteristics of the participants are presented in Table 2. The percentage of male patients with lung cancer is significantly higher than that in females, with 67.5% of men and 32.5% of women, with obvious differences. Therefore, in the age distribution, it was found that the elderly have a high incidence of lung cancer, and the people under 60 years of age accounted for only 21.8%. However, there is no obvious difference in the season of onset. Generally speaking, there are more patients in spring, and the number of patients in autumn is relatively small.

Through the distribution of the spatial form in the study area (Figure 2(a)), we used ArcGIS software to analyse the spatial distribution of lung cancer patients from 2014 to 2020 and calculate the density of lung cancer patients in the study area in units, which can directly reflect the distribution of lung cancer patients in the study area. The results showed that the lung cancer patients were clustered in units YH07 and YH08 (Figure 2(b)).

### 4.2. Analysis of Factors Influencing the Development of Lung Cancer

The results of Spearman's rank correlation analysis showed that land use, road transport, spatial form, green space and open space, service facilities, and natural environment were all related to the incidence of lung cancer (*P* < 0.05), and there was no correlation between the annual mean NO_2_ and the annual mean O_3_ (*P* > 0.05) (Table 3).

#### 4.2.1. Built Environment

In terms of the built environment, according to Spearman's rank correlation model, residential density was significantly positively correlated with the incidence of lung cancer, with a correlation coefficient of 0.099, which indicates that the increasing residential density increases the risk of developing lung cancer. In addition, the distance to industry had a significant negative correlation with the incidence of lung cancer, with a correlation coefficient of −0.075, and this suggests that the risk of lung cancer tends to increase the closer you are to industrial area.

In terms of road traffic, there was a significant positive correlation between lung cancer incidence and traffic density and road intersection density, and the correlation coefficients were 0.143 and 0.148respectively. Therefore, the risk of lung cancer tends to increase when road density increases with road intersection density. In addition, there was a significant positive correlation between the bus stop density and the incidence of lung cancer within the 500 m buffer zone, with a correlation coefficient of 0.230. This indicates that an increase in bus stop density increases the incidence of lung cancer. The distance between the residents and main roads was negatively correlated with the incidence of lung cancer with a correlation coefficient of −0.090. It shows that a closer distance from the main road tends to increase the incidence of lung cancer.

The model showed that the building density was of a significant positive correlation with the incidence of lung cancer, with a correlation coefficient of 0.120. Therefore, the incidence of lung cancer tends to increase with increasing building density. Moreover, there was a significant positive correlation between the FAR and the incidence of lung cancer, with a correlation coefficient of 0.135, and this indicates that the incidence of lung cancer tends to increase with higher FAR. In addition, according to the results of the model, the Normalized Difference Vegetation Index (NDVI) showed a significant negative correlation with the incidence of lung cancer, with a correlation coefficient of −0.142. It indicates that the incidence of lung cancer tends to decrease with higher NDVI. In addition, the distance to the river had a significant positive correlation with the incidence of lung cancer, with a correlation coefficient of 0.162. Therefore, proximity to rivers tends to reduce the incidence of lung cancer. The distance to the park was negatively correlated with the incidence of lung cancer, with a correlation coefficient of −0.121. It indicates that the proximity to parks tends to increase the incidence of lung cancer.

In terms of service facilities, the model showed that the cigarette and wine shops' density within the 500 m buffer zone was significantly positively correlated with the incidence of lung cancer, with a correlation coefficient of 0.290. Therefore, lung cancer incidence tends to increase when the cigarette and wine shops density increases. In addition, food and beverage density within the 500 m buffer zone showed a significant positive correlation with the incidence of lung cancer, with a correlation coefficient of 0.269, and it is suggested that the greater the density of food and beverage, the higher the incidence of lung cancer tends to increase.

#### 4.2.2. Natural Environment

In terms of the natural environment, according to the model, the annual average PM_2.5_, PM_10_, and SO_2_ were significantly positively correlated with the incidence of lung cancer, and the correlation coefficients were 0.073, 0.170, and 0.162, respectively. Therefore, lung cancer incidence tends to increase with increasing concentrations of particulate matter pollution. And average CO was significantly positively correlated with the incidence of lung cancer, with a correlation coefficient of 0.170. This indicates that the incidence of lung cancer tends to increase with increasing gaseous pollutants concentration. Meanwhile, the annual average NO_2_ and O_3_ were not strongly correlated with the incidence of lung cancer.

### 4.3. Analysis of Geographical Detector Results

Through Spearman's rank correlation, we further extracted ten built-environment and natural-environment indexes and used the geographic detector to study the impact of the urban environment on the incidence of lung cancer. In the test of factors affecting the lung cancer incidence through 2014–2020, we found that all of the indicators passed the significance test (*P* < 0.05), and the higher the *q* value, the greater the impact (Figure 3). We found that road intersections density and the distance to industry accounted for more than 10% of the lung cancer risk, with FAR, SO_2_, PM_10_, distance to the river, cigarette and wine shop density, distance to the main road, and bus stop density accounting for more than 1% of the lung cancer risk, is a secondary factor. This indicates that road intersection density and the distance to the industry are the main factors influencing the risk of lung cancer.

On a seasonal scale, we found that the effect of the index factors on the lung cancer patients was different in different seasons (Figure 3). Spring is mainly affected by road intersection density, distance to industry, SO_2_, cigarette and wine shop density, distance to main road, PM_10_, distance to river, and FAR. Summer is mainly affected by road intersection density, distance to industry, and FAR. Autumn is mainly influenced by road intersection density and the distance to industry. Winter is mainly affected by road intersection density, distance to the industry, FAR, distance to the river, SO_2_, and PM_10_. On the whole, road intersection density and the distance to industry were the common influence factors of each quarter, and the *q* value was higher. While the environmental indicators of different quarters had different effects and the influence of spring and winter was greater, the environmental impact is relatively small in summer and autumn. The study found that older people, as well as men, are usually more pronounced to seasonal changes [22] and that the study area has more older people who are more susceptible to seasonal changes. And with spring and winter likely to increase PM_2.5_ concentrations and a more polluted environment [23], the risk of developing lung cancer may be relatively higher.

The incidence of lung cancer is affected by the city environment. The risk of lung cancer is not only a single factor, but also the interaction of environmental factors may increase or decrease the influence of individual factors. Through the interaction analysis of environmental indicator factors for 2014–2020 (Figure 4), we found that both interactions of independent variables played an enhanced role at the annual scale. The strongest interaction was found between cigarette and wine shop density and road intersection density (*q* = 0.30). This was followed by the distance to industry and the distance to the river (*q* = 0.27), followed closely by food and beverage density and road intersection density (*q* = 0.26).

On the quarterly scale, the interaction of all environmental indicators is enhanced and the *q* value of the interaction is increased compared with that of the single environmental indicator (Figure 4). In spring, the strongest interaction was between road intersection density and cigarette and wine shop density (*q* = 0.56), followed by the interaction between the distance to industry and PM_10_ (*q* = 0.49), and the distance to industry and SO_2_ (*q* = 0.48). In summer, the strongest interaction was between road intersection density and the distance to industry (*q* = 0.23). The interaction between road intersection density and the distance to industry had the strongest effect in autumn (*q* = 0.50). In winter, the strongest interaction was between road intersection density and the distance to industry, distance to river, SO_2,_ and PM_10_ (*q* = 0.26).

Overall, there were more interactive influences on the lung cancer incidence in spring and winter and fewer interactive elements in summer and autumn. In addition, road intersection density and the distance to industry were the main risk factors interacting with the incidence of lung cancer.

## 5. Discussion

This study analysed the basic characteristics of the population with lung cancer disease and examined the correlation between the different influences of the urban environment and the incidence of lung cancer by using Spearman's rank correlation model. The interaction of each indicator was analysed using a geographic detector model and an enhanced effect of two-by-two interactions between the indicators was found. Thus, effective strategies are provided for urban development to reduce the risk of lung cancer incidence.

According to the analysis of the distribution characteristics of the lung cancer incidence, it was found that the main population of the lung cancer incidence is male, and the incidence of middle-aged and old people is higher, which is consistent with the international research [24]. The existing studies have demonstrated that genes (family history) and living habits (smoking, second-hand smoke, and kitchen smoke) contribute to the risk of lung cancer [25, 26]. Tobacco is an important risk factor for tumours and the prevalence of smoking is generally higher in Chinese men than in women [27], which may explain the higher incidence of lung cancer in men than in women. And the study found that 61% of women who died of lung cancer were nonsmokers. The decline in smoking rates among Chinese women has been accompanied by an increase in lung cancer [28], suggesting that the risk factors contributing to the development of lung cancer are unclear.

Studies have found that in the built environment, different land use properties have different effects on respiratory disease [29], consistent with the studies that the residential density has a significant positive effect on lung cancer incidence, the distance to industry is a negative effect, and road traffic density has a significant positive effect on the lung cancer incidence. Urban construction sites can have an impact on air quality in cities [30], with excessive residential density being detrimental to residential ventilation and increasing pollutant exposure. In factor detection, we found that the distance to industry and road intersection density were the main influencing factors for lung cancer incidence in the population in four seasons, and the interaction of the distance to industry and road intersection density significantly enhanced the risk of lung cancer incidence in the population. The density of roads and intersections reflects the volume of traffic to a certain extent, and the higher the density, the higher the incidence rate [31], and according to the foreign studies, male residents living in areas with more motor vehicles have a higher risk of cancer [32], while Sinharay's latest invention study published in the Lancet shows that vehicle emissions have a negative impact on the cardiopulmonary function of the population [33]. And industrial emissions increase atmospheric pollution, and studies have proven that particulate pollution is an important cause of respiratory disease [34]; so, long-term exposure to pollutant gases increases the risk of lung cancer. Meanwhile, the spatial form has a significant positive effect on lung cancer incidence, and an increase in building density and FAR also increases the incidence of lung cancer. Excessive building density and FAR lead to high population density, reduce greenery quality, increase air pollution exposure, affect urban ventilation, raise the risk of lung cancer incidence, and increase the risk of death of lung cancer patients [35].

The bus stop density has a significant positive influence on the incidence of lung cancer. It has been found in the studies that the longer waiting time at the bus stop will cause longer exposure to air pollutants, leading to a higher risk of respiratory diseases [36, 37], and some studies have suggested that bus stops could enhance accessibility and community social network and increase residents' physical activity [38], so as to effectively reduce the risk of respiratory diseases; moreover, it is also conducive to the daily activities of the elderly, thus effectively providing the daily activity space for the elderly and a guideline for a healthy lifestyle [39]. The results of this study show that higher bus stop density will contribute to the higher incidence of lung cancer, for which the reason may be that public transportation serves as the main mode of traffic travel in the study area, and the bus stops are always established at the places with higher population density and the aggregation places of elderly population, and the elderly are more susceptible to the influence of the built environment [40], so more bus stops will increase the crowd gathering risk and increase the exposure to environmental pollution while providing convenient transportation.

In line with the previous studies, we found that NDVI has a significant negative impact on the lung cancer incidence, while the distance to the river has a significant positive impact. Vegetation coverage and rivers can reduce pollutant concentration [41]. According to the research between the green space and health, it is found that planting 11 trees more in an urban block can reduce the cardio-metabolic status and the incidence of respiratory diseases [42], and water can reduce air pollution and the risk of exposure to pollutants [43]. People who engage in more physical activity have a significantly lower risk of developing diseases such as lung cancer, according to study finds [44], and physical activities may reduce the risk of lung cancer in current or former female smokers [45]. Friedenreich found that leisure physical activities could better reduce the risk of lung cancer than occupational physical activities [46]. This suggests that the physical activity is effective in reducing the risk of lung cancer, and that areas with high vegetation cover and proximity to rivers can attract people to increase their physical activity.

However, it is interesting to note that the closer we are to the park, the higher the incidence of lung cancer tends to be. Previous studies have found that the open green space can increase the physical activity, create good space, reduce air pollution, and reduce respiratory diseases [47, 48], but other studies have found no significant correlation between urban green space and lung cancer mortality, road greening, and virescence in front of houses can increase the rate of green space, but cannot provide people with recreation [49], while the community park and the amusement park are the important places of high-frequency physical activity [50]. Considering that the study area is located in the old city, the study population is mainly elderly, densely populated, with high building density, and the park open space is mainly Zhanggongshan Park, and the population is concentrated near the park and has a high incidence of lung cancer.

There is a significant positive correlation between the POI points of service facilities around the residential areas and the incidence of lung cancer, which is consistent with the general studies. The daily activity distance that can meet the basic material and life needs of the residents by 10-min walking is 500 m [51]. The results show that smoking and drinking constitute one of the main causes of lung cancer [52]; therefore, the larger number of cigarette and wine shops in the vicinity of residential areas will provide higher convenience for the residents, which will indirectly increase the risk of lung cancer. And we found a higher q value for the interaction between intersection density and tobacco shops, indicating that the more tobacco shops near an intersection, the higher the risk of people developing lung cancer, and that public services should be allocated appropriately. Too many restaurants around the residential areas will increase the emission of cooking fumes, thereby increasing PM_2.5_ concentration in the air and leading to an increase in the incidence of lung cancer [53]. A lot of grease and sewage drainage in restaurants will also impair the respiratory system. In addition, the increase of automobile service facilities around the residential areas will increase the traffic load, and the centralized parking facilities, gas stations, and other facilities will easily lead to the agglomeration of vehicles and heavier automobile exhaust, thereby causing air pollution and increasing the incidence of lung cancer [54].

In terms of the natural environment, we have found that air pollution has a positive effect on the incidence of lung cancer, and that air pollution is one of the greatest threats to the health of the population, with air pollution increasing the incidence of respiratory diseases [55]. Studies have concluded that solid-particulate matter pollution in the atmosphere has a significant effect on lung cancer incidence. A study of urban areas in Shanghai found that for every 10 *μ*g/m^3^ increase in atmospheric SO_2_ concentration, the number of total deaths, cardiovascular deaths, and respiratory deaths in the urban areas of Shanghai increased by 1.25%, 1.45%, and 1.71%, respectively [56]. The increase in average daily CO increases the risk of outpatient visits for respiratory diseases and has a higher impact on women and elderly patients [57], who are more vulnerable to air pollution than younger people [58, 59]. High concentrations of particulate matter (PM) are an important risk factor for respiratory diseases, especially near industrial areas, which increase particulate matter concentrations, and PM_2.5_ concentrations are generally higher in winter [60].

## 6. Conclusion and Suggestions

### 6.1. Conclusion

This study provides a multilevel model based on the impact of urban multiple environmental factors on lung cancer and explores the characteristics of urban multiple environmental factors significantly related to lung cancer, and the correlation (*P* value <0.05) is statistically significant. We have come to the following conclusions: (1) Through spatial distribution analysis, it is found that there are significant differences in the incidence of lung cancer. The main population groups affected by lung cancer are concentrated in the over 60s and men. And the population with lung cancer is clustered concentrated in the vicinity of Zhanggongshan Park. (2) Under the analysis of model construction, the urban environment has a significant impact on the incidence of lung cancer, among which land use, road traffic, spatial form, green space and open space, air pollution, and service facilities have significant correlations with the incidence of lung cancer. (3) Factor detection and interaction analysis revealed a greater effect of spring and winter on lung cancer prevalence. The road intersection density and the distance to the industrial area are the most important potential influencing factors, and the interaction of any two factors will increase the risk of lung cancer. Therefore, it is necessary to take reasonable measures to reduce the risk of lung cancer.

### 6.2. Suggestions

#### 6.2.1. Improve the Spatial Layout

Focus on the layout of the urban space, improve public service facilities, and enhance urban management and governance. Improve residential quality, reduce building density, increase open space, optimise the urban spatial system, and provide a comfortable and pleasant living environment. In terms of industrial layout, polluting industrial sites should be located away from urban areas and nonpolluting industries should be combined with the construction of central areas of the city, where population density is high and increasing industries can increase employment opportunities, thereby reducing the use of motor vehicles and lowering air pollution.

#### 6.2.2. Optimize Road System

Improving the road network system, optimising the shape of the neighbourhood, enhancing street connectivity, and improving the neighbourhood environment can effectively increase accessibility and improve the mobility of people. The pedestrianised streets are increased and the neighbourhood form is constructed in a “small neighbourhood, dense road network” layout. Reducing the traffic capacity of the sites around residential areas, optimising the road environment, reducing the rate of car travel, increasing the rate of walking and cycling, reducing the exposure of residents to high concentrations of motor vehicle emissions, and limiting traffic at road junctions with poor air quality will help to improve the urban environment.

#### 6.2.3. Increase Green Space and Open Space

Air pollution is an important risk factor for respiratory diseases. Therefore, the effective reduction of air pollution can effectively prevent respiratory diseases. And a large number of green spaces can absorb particulate pollution and reduce exposure to pollutants, and large areas of water can alleviate air pollution and can reduce the distribution of particulate matter. Therefore, to create a good environment scene, enhance air circulation, is conducive to increase the physical activity of residents, effective prevention of respiratory diseases, and promoting physical health.

The study mainly analysed the distribution characteristics of lung cancer patients from 2014 to 2020 and explored the influence of the multifactor environmental influence mechanism on the lung cancer patients, and through the analysis of its correlation and interaction, it can provide some references for the pathogenesis of lung cancer and make a little contribution for the future research and development. This study is mainly in the old industrial area of the study area; there is no focus on the analysis of the impact of industrial change on the incidence of lung cancer, but in the model establishment research, because of the reason that the data did not add the patient's own habit and lifestyle influence, this may take the later stage more thorough research.

## Figures and Tables

**Figure 1:** The location of old town, Bengbu, China.

**Figure 2:** Spatial form distribution and the spatial distribution of lung cancer incidence population in the old town of Bengbu city, 2014–2020.

**Figure 3:** Annual and seasonal scale factor detection in the old urban areas of Bengbu City, China, 2014–2020. Note: In spring, road intersection density, distance to industry, SO_2_, cigarette and wine shop density, distance to the main road, PM_10_, distance to the river, and FAR were significant (*P* < 0.05); in summer, road intersection density and the distance to industry were significant (*P* < 0.05); in autumn, road intersection density and distance to industry were significant (*P* < 0.05); in winter, road intersection density, FAR, distance to industry, SO_2_, and PM_10_ were significant (*P* < 0.05).

**Figure 4:** Annual and seasonal independent variable interaction detection. Note: DTR represents the distance to the river, DTI represents the distance to industry, DTMR represents the distance to the main road, BSD represents bus stop density, RID represents road intersections density, FABD represents food and beverage density, CAWSD represents cigarette and wine shop density, FAR represents the floor-area ratio, PM_2.5_ represents the concentration of PM_2.5_, PM_10_ represents the concentration of PM_10_, and SO_2_ represents the concentration of SO_2._.

**Table 1:** A system of environmental impact factors on lung cancer incidence in the study area of Bengbu, China.

Environmental factors	Categories	Subcategories	Specific variables	Unit
Built environment	Land use	Residential density	Residential patch density	%
		Distance to industry	The shortest distance from industrial land	m
	Road traffic	Traffic density	Total road density	pcs/ha
		Distance to main road	Distance from the nearest main road	pcs/ha
		Road intersection density	Intersection density, the number of road intersections in 500 m buffer zone	pcs/ha
		Bus stops density	Bus station density, the number of bus stops in 500 m buffer zone	pcs/ha
	Spatial form	Building density	Building coverage, the building base area/total land area	%
		Volume fraction	Total construction area/total land area	—
	Green space and open space	Vegetation cover	Normalized Difference Vegetation Index (NDVI)	—
		Distance to river	Distance from the nearest river	m
		Distance to park	Distance from the nearest open activity space	m
	Service facility	Cigarette and wine shop density	Number of tobacco and liquor stores in 500 m buffer zone/buffer zone area	pcs/ha
		Food and beverage density	Number of catering facilities in 500 m buffer zone/buffer zone area	pcs/ha

**Table 2:** Analysis of basic characteristics of lung cancer incidence population in the old town of Bengbu city from 2014 to 2020.

Variables	Classification	Number of cases	Proportion of patients (%)
Gender	Man	303	67.5
	Woman	146	32.5

Age	≥60-years-old	351	78.2
	<60-years-old	98	21.8

Dead season	Spring (March–May)	114	25.4
	Summer (June–August)	121	26.9
	Autumn (September–November)	100	22.3
	Winter (December–February of the following year)	114	25.4

**Table 3:** Relationship between Spearman's rank correlation test independent variables and the incidence of lung cancer in the old town of Bengbu city, China.

Environment factors	Categories	Subcategories	Variables	Correlation coefficient	Sig.(two-side)
Built environment	Land use	Residential density	Residential patch density	0.099^*∗∗*^	0.001
		Distance to industry	Distance from the nearest industry	−0.075^*∗*^	0.014
	Road traffic	Traffic density	Road network density	0.143^*∗∗*^	0.000
		Road intersection density	Road intersection density in 500 m buffer zone	0.148^*∗∗*^	0.000
		Distance to the main road	Distance from the nearest trunk road	−0.090^*∗∗*^	0.003
		Bus stop density	Density of bus stops in 500 m buffer zone	0.230^*∗∗*^	0.000
	Spatial form	Building density	Building coverage	0.120^*∗∗*^	0.000
		FAR (floor-area ratio)	Floor-area ratio	0.135^*∗∗*^	0.000
	Green space and open space	NDVI	Normalized Difference Vegetation Index (NDVI) in January	−0.142^*∗∗*^	0.000
		Distance to river	Distance from the nearest river	0.162^*∗∗*^	0.000
		Distance to park	Distance from the nearest open space	−0.121^*∗∗*^	0.000
	Service facility	Cigarette and wine shop density	Number of tobacco and liquor stores in 500 m buffer zone	0.290^*∗∗*^	0.000
		Food and beverage density	Food and beverage quantity in 500 m buffer zone	0.269^*∗∗*^	0.000

Natural environment	Air pollution	Particulate matter (PM) concentration	Average mean PM_2.5_	0.073^*∗*^	0.018
			Average mean PM_10_	0.170^*∗∗*^	0.000
			Average mean SO_2_	0.162^*∗∗*^	0.000
		Gaseous pollutants concentration	Average mean NO_2_	0.020	0.512
			Average mean O_3_	0.034	0.270
			Average mean CO	0.170^*∗∗*^	0.000

Note. ^*∗*^*P* < 0.05, ^*∗∗*^*P* < 0.01.

## Data Availability

The datasets generated and/or analysed during the current study are not publicly available but are available from the corresponding author on a reasonable request.
